The article "Decreased expression of miR-939 contributes to chemoresistance and metastasis of gastric cancer via dysregulation of SLC34A2 and Raf/MEK/ERK pathway" was retracted in 2022. Reasons: duplicated images; unreliable data; concerns about the data; concerns about the images.

# Decreased expression of miR-939 contributes to chemoresistance and metastasis of gastric cancer via dysregulation of SLC34A2 and Raf/MEK/ERK pathway

**DOI:** 10.1186/s12943-017-0586-y

**Published:** 2017-01-23

**Authors:** Jia-Xing Zhang, Yi Xu, Ying Gao, Cui Chen, Zhou-San Zheng, Miao Yun, Hui-Wen Weng, Dan Xie, Sheng Ye

**Affiliations:** 1 Department of Oncology, the First Affiliated Hospital, Sun Yat-sen University, No. 58, Zhongshan road II, 510080 Guangzhou, People’s Republic of China; 2 The State Key Laboratory of Oncology in South China, Sun Yat-Sen University Cancer Center, Collaborative Innovation Center for Cancer Medicine, No. 651, Dongfeng Road East, 510060 Guangzhou, People’s Republic of China; 3 Department of Pathology, Sun Yat-Sen University Cancer Center, Guangzhou, People’s Republic of China

**Keywords:** miR-939, SLC34A2, Gastric cancer, Chemoresistance, Metastasis

## Abstract

**Background:**

The development of chemoresistance and metastasis are the leading causes of death for gastric cancer (GC) patients, however, the molecular mechanisms involved remain unclear. Dysregulation of miRNAs is associated with a variety of disease, including GC. Recently, microarray profiling analysis revealed that miR-939 was dysregulated in human GC samples, but the role of miR-939 in GC has not been intensively investigated.

**Methods:**

In the present study, we firstly examined the expression pattern of miR-939 in two independent cohorts of clinical GC samples: one cohort of 112 GC patients with stage I-III disease who underwent surgery followed by adjuvant chemotherapy; and another cohort of 110 GC patients with stage IV disease who received palliative chemotherapy. A series of in vivo and in vitro assays were then performed to investigate the function of miR-939 in GC.

**Results:**

We detected that reduced expression of miR-939 was associated with chemoresistance and increased risk of tumor recurrence in GC patients. Further function study demonstrated that overexpression of miR-939 suppressed GC cell growth, and enhanced 5-fluorouracil-induced chemosensitivity by compromising cellular growth and inducing apoptosis in vitro and in vivo. Moreover, miR-939 repressed the migration and invasion of GC cells in vitro, and diminished the occurrence of lung metastasis in vivo. We further identified solute carrier family 34 member 2 (SLC34A2) was a novel target of miR-939. Mechanistically, we elucidated that miR-939 exerted its function mainly through inhibiting SLC34A2/Raf/MEK/ERK pathway, which is activated in GC. Multivariate analysis identified miR-939, SLC34A2, and their combination as independent indicators for poor prognosis and tumor recurrence in GC patients.

**Conclusion:**

Our data indicate that miR-939 acts as a tumor suppressor miRNA in GC, and miR-939/SLC34A2 axis represents a novel therapeutic strategy for future GC treatment.

**Electronic supplementary material:**

The online version of this article (doi:10.1186/s12943-017-0586-y) contains supplementary material, which is available to authorized users.

## Background

Gastric cancer (GC) is one of the most common causes of cancer-related deaths worldwide [1]. At present, surgical resection and palliative chemotherapy are the backbone treatment modalities for early staged and advanced staged GC patients, respectively [2]. Although tremendous progress has been made in therapeutic strategies, the prognosis for GC patients using existing treatments remains unsatisfactory. The development of chemoresistance and metastasis are the leading causes of death for GC patients, however, the molecular mechanisms involved remain unclear [3–5]. Therefore, a better understanding of these molecular events will undoubtedly facilitate our ability to the development of novel therapeutic targets and strategies for GC treatment.

MicroRNAs (miRNAs) are a class of small-regulatory RNA molecules that repress protein translation through binding to the 3’-untranlated region (UTR) of their target mRNA [6]. Aberrant expression of miRNAs has been reported in various types of cancers [7, 8]. In GC, miR-192, miR-215, miR-25 are reported to be upregulated, whereas miR-375, miR-101 are downregulated [9–12]. Nevertheless, the role of miRNAs in the regulation of GC-associated genes, and thus the role of miRNAs in the pathogenesis of GC, remains elusive.

Recently, microarray profiling analysis revealed that a number of miRNAs were dysregulated in human GC samples compared with normal tissues, including miR-939 [13]. However, the clinical significance and biological role of miR-939 in GC is still not known. Therefore, we devised our present study to find out the mechanism of miR-939 action and its potential clinical application in GC. Interestingly, we found that decreased miR-939 expression is closely related with poor clinical outcome of GC patients. Our data showed that miR-939 inhibits GC metastasis and enhances the sensitivity of GC cells to 5-fluorouracil (5-Fu) treatment. In addition, we identified that miR-939 exerts its tumor-suppressing role by targeting SLC34A2 via the inhibition of Raf-MEK-ERK signaling pathways.

## Methods

### Cell lines

Gastric cancer cell lines (AGS, BGC-823, HGC-27, MGC-803, MNK-45, and SGC-7901), and one immortalized human gastric epithelial mucosa cell line (GES-1) were grown in DMEM medium supplemented with 10% fetal bovine serum.

### Samples and patients

For the use of clinical materials for research purposes, prior approval was obtained form the Committees for Ethical Review of Research at Sun Yat-Sen University (Guangzhou, China). Formalin-fixed paraffin-embedded (FFPE) tumorous and adjacent non-tumorous tissues samples from 112 GC patients, who underwent surgical resection between January 2010 and December 2011, were randomly selected from the archives of the Department of Pathology of Sun Yat-Sen University Cancer Center (Guangzhou, China). All the patients enrolled were diagnosed with stage I-III GC disease during surgery resection, and received postoperative adjuvant 5-Fu-based chemotherapy: SOX regimen (Tegafur plus oxaliplatin), XELOX regimen (capecitabine plus oxaliplatin), Tegafur, or capecitabine. The clinicopathological characteristics of the patients in this cohort are summarized in Additional file 1: Table S1. The patients were followed every 3 months for the first year and then every 6 months for the next 2 years, and finally annually, thereafter. The diagnostic examinations consisted of CT, MRI, abdominal ultrasonography and bone scan when necessary to detect recurrence and/or metastasis. During follow-up period, 48 patients experienced tumor recurrence or metastasis, and 38 deaths due to cancer-related diseases.

In addition, we obtained another independent cohort of 110 patients, who were diagnosed with stage IV GC disease between January 2008 and December 2013. The mean age at diagnosis was 56 years (range, 21–81 years); 72 patients were male. The patients in this cohort were administrated with fluorouracil-based regimen (SOX or XELOX) as first-line palliative chemotherapy. The response of chemotherapy was assessed based on CT examination every 6 weeks during therapy and at the end of treatment according to the following criteria: complete response (CR) as defined by the complete resolution of all assessable lesions; partial response (PR) as defined by a reduction by 50% or more of the sum of the lesions and no progression of assessable lesions; or no change (NC) as indicated by a reduction <50% or increase <25% in tumor size. The CR, PR or NC conditions had to last for at least 4 weeks without appearance of new lesions. Otherwise the response will be counted as progressive disease (PD) as defined by an increase of 25% in tumor size or appearance of new lesions.

The clinical and clinicopathological classification and stage were determined according to the American Joint Committee on Cancer (AJCC) criteria. Patients who had a single primary lesion without neoadjuvant therapy before operation were included in the study. Other criteria for inclusion were as follows: age >18 years; histologically confirmed gastric cancer with at least one measurable lesion as defined by the Response Evaluation Criteria in Solid Tumors; Eastern Cooperative Oncology Group performance status (ECOG PS) of B2, and life expectancy >3 months.

For both XELOX and SOX regimen, oxaliplatin (130 mg/m2) was diluted in 500 mL of 5% dextrose and infused intravenously over 2 h on day 1. Oral administration of capecitabine (1000 mg/m2) and Tegafur (body surface area, BSA < 1.25: 40 mg; BSA 1.25–1.5: 50 mg; BSA > 1.5: 60 mg) was followed twice a day from days 2 to 15 in XELOX and SOX regimen, respectively. Treatment was continued until 6–8 cycles of XELOX, SOX, Tegafur, or capecitabine had been completed, disease progression, unacceptable toxicity, patient withdrawal, or physician’s decision.

### RNA isolation and quantitative real-time PCR

Total RNA was extracted from cultured cells and tissue specimens using TRIzol (Invitrogen, Calsbad, CA). Real-time PCR was carried out with SYBR Green SuperMix (Roche, Basel, Switzerland) using ABI7900HT Fast Real- Time PCR system (Applied Biosystems, Foster City, CA). Glyceraldehyde-3-phosphate dehydrogenase (GAPDH) or U6 was used as an internal control. An optimal cutoff value for “high” or “low” miR-939 expression was identified based on the median value of the cohorts of patients tested. TaqMan probes were used to detect miR-939, SLC34A2, U6, and GAPDH (GeneCopoeia, Guangzhou, China).

### MTT assay

Cell viability was measured by a 3-(4, 5-dimethylthiazol-2-yl)-2, 5-diphenyl tetrazolium bromide (MTT) assay (Sigma, St, Louis, Missouri, USA). Briefly, cells were seeded in 96-well plates and treated with various concentration of 5-Fu for each well. The absorbance was measured at 570 nm, with 655 nm as the reference wavelength. All experiments were carried out in triplicates.

### Colony formation assay

Cells were placed in six-well plate (500 cells/plate) and cultured for 2 weeks. Colonies were fixed with methanol for 5 min, and stained with 0.1% crystal violet for 30 s.

### Flow cytometric analysis of apoptosis

Annexin V-APC and propidium iodide (PI) stains were carried out to assess the percentage of cells undergoing apoptosis. The apoptosis assay was conducted using the protocol supplied by the manufacturer (BioVision Inc.). Each sample was then subjected to analyses by flow cytometry (Beckman Coulter, cytomics FC 500, CA).

### Wound-healing, migration and invasion assays

For cell would-healing assay, the movement of cells was measured in a scraped, acellular area made by a 200 ml pipette tube, and the spread of wound closure was observed after 24 h. For migration assay, 40,000 cells were added to the upper chamber in serum free media and migration at 37 °C towards 10% FBS containing growth media was determined either after 24 h. Cells migrated through the membrane were fixed, stained and counted under light microscope. For invasion assays, 1 × 10^5^ cells were seeded into a Matrigel invasion chamber (BD Biosciences, NJ, USA) in a 24-well culture plate. After 24 h, the invasive cells located on the lower side of the chamber were fixed in methanal, stained with crystal violet, and followed by counting under a light microscope.

### Western blot (WB) assay

Equal amounts of cell protein lysates were resolved by SDS-polyacrylamidegel electrophoresis (PAGE) and electrotransferred on a polyvinylidene difluoride (PVDF) membrane (Pall Corp., Port Washington, NY) according to standard methods. The following primary antibodies were used: anti-SLC34A2 (Abcam, Cambridge, UK); anti-GAPDH, anti-AKT, anti-p-AKT, anti-ERK, anti-p-ERK, anti-c-Raf (Cell signaling Technology, Beverly, MA).

### Immunohistochemical (IHC) Staining

In brief, tissue sections were de-waxed and incubated in retrieval buffer solution for antigen recovery. We used the Dako Real Envision Kit (K5007, Dako) to visualize protein expression after staining with primary antibody. Staining intensity was scored manually by two independent experienced pathologists as 0 = no staining, 1 = weak staining, 2 = moderate staining, and 3 = strong staining. Tumor cells in five fields were randomly selected and scored based on the percentage of positively stained cells (0–100%). The final IHC score was calculated by multiplying the intensity score with the percentage of positive cells (range from 0 to 3). An optimal cutoff value was identified based on the median value of the cohorts of patients test.

### Vector construction and retroviral infection

The miR-939 expression vector (HmiR0533-MR03), the control vector for miR-939 (CmiR0001-MR03), the coding sequences of SLC34A2 expression vector (EX-A3175-Lv105), and the control vector for SLC34A2 (EX-NEG-Lv105) were purchased from the GeneCopoeia Company (Guangzhou, China). Cells transfected with empty vector were used as controls. The vectors were packaged using the ViraPower Mix (Genecopoeia, Guangzhou, China) in 293FT cells. After culturing for 48 h, the lentiviral particles in the supernatant were harvested and filtered by centrifugation at 500 *g* for 10 min, and then transfected into the GC cells.

### Mimic, antagomir, plasmids and transient transfection

miR-939 mimic and antagomir-939 were purchased from GeneCopoeia Company (GuangZhou, China). Oligonucleotide transfection was performed with Lipofectamine 2000 reagent (Invitrogen, Carlsbad, CA), according to the manufacturer’s instructions.

### Luciferase reporter assay

The 3′ UTR of SLC34A2 were amplified and cloned downstream to the luciferase gene in a modified pGL3 control vector. The firefly luciferase construct was cotransfected with a control Renilla luciferase vector into GC cells in the presence of miR-939 mimic, antagomir-939, or miR-control. A dual luciferase assay (Promega) was performed 48 h after transfection. The experiments were performed independently in triplicate.

### Animal experiments

For in vivo metastasis assays,six Four-week-old BALB/c nude mice in each experimental group were injected with SGC-7901/control or SGC-7901/miR-939 cells, respectively. Briefly, 2 × 10^5^ GC cells in 30 μl of 33% Matrigel (Becton Dickinson, NJ, USA) were injected intravenously through the tail vein. The experiment was terminated 28 days after tumor-cell inoculation, and metastatic nodules in each lung were counted.

For xenograft growth of orthotopic animal model assay, the mice were randomly divided into four groups (*n* = 6): SGC-7901/control, SGC-7901/miR-939, SGC-7901/control + 5-Fu, SGC-7901/miR-939 + 5-Fu, and equal amounts of SGC-7901/miR-939 or SGC-7901/control cells (3 × 10^6^) were injected subcutanesouly into the flank of each mouse. For chemotherapy treatment group: 5-Fu was administered at a dose of 5 mg/kg at 10 am twice a week for 3 week; for control groups, DMSO alone (100% DMSO, 40 lL, intraperitoneal injection every 2 days) was delivered to the mice. Treatment began on day 7, when the tumors were measurable. The tumors were examined twice weekly, length and width measurements were obtained with calipers, and the tumor volumes were calculated. On day 25, the animals were euthanized and the tumors were excised and weighed.

All the procedures were carried out in accordance with the guidelines of the Laboratory Animal Ethics Committee of Sun Yat-Sen University.

### Statistical analysis

Statistical analysis was performed using a SPSS software package (SPSS Standard version 16.0, SPSS Inc). Receiver operating characteristic (ROC) curve analysis was conducted to evaluate the predictive value of miR-939 expression in predicting GC chemotherapy response. Comparisons between groups for statistical significance were performed with a 2-tailed Student’s *t* test. Bivariate correlations between study variables were calculated by Pearson’s correlation coefficients. Differences between variables were assessed by the Chi-square test or Fisher’s exact test. For survival analysis, we analyzed all GC patients by Kaplane-Meier analysis. A log rank test was used to compare different survival curves. Multivariate survival analysis was performed on all parameters that were found to be significant in univariate analysis using the Cox regression model. *P* values <0.05 were considered significant.

## Results

### Expression of miR-939 is downregulated in GC and closely related to clinical outcomes

To explore miR-939 expression in GC, we conducted real-time PCR assay. As shown in Fig. 1a, b, the expression of miR-939 was significantly decreased in human GC cell lines and human primary GC tissues compared with normal gastric epithelial cell lines and nontumor human gastric tissues, respectively (*P* < 0.05).

**Fig. 1:** miR-939 is down-regulated in gastric cancer tissues and cell lines, and inhibits GC proliferation. **a** comparison miR-939 expression in six GC cell lines and non-transformed epithelial cell line, GES-1. **b** comparing differences in the expression levels of miR-939 between tumor and corresponding non-tumor tissues. **c** comparing differences in the expression levels of miR-939 between GC tumor tissues from recurrent and non-recurrent patients. **d** the predictive value of miR-939 expression regarding the chemotherapy response in 110 patients with advanced GC disease. ROC curve analysis for miR-939 expression was performed to assess GC treatment response (area under the curve [AUC] = 0.777, *P* < 0.001). **e** and **f** MTT assays (**e**) and colony formation assay (**f**) indicate that the proliferation and tumorigenicity of miR-939-overexpressing cells was decreased, and that of the miR-939-silenced cells was increased, compared with control cells. Expression levels of miR-939 were determined by qRT-PCR and normalized against an endogenous control (U6 RNA). *P < 0.05, ** *P* < 0.01

Next, we analyzed miR-939 expression using pretreatment tissue specimens from 112 GC patients with stage I-III disease who underwent surgery resection followed by adjuvant chemotherapy. We detected that miR-939 levels were significantly decreased in patients who showed local relapse or distant metastasis in comparison to patients who did not have tumor relapse or metastasis during our follow-up period (*P* < 0.05,Fig. 1c).

To further determine the clinical implication of miR-939 expression, we conducted qRT-PCR assay in 110 pretreatment samples from stage IV GC patients who received palliative chemotherapy. Among the enrolled cases, there were 0, 57, 36, and 17 patients satisfied the criteria for complete response (CR), partial response (PR), no change (NC) and progressive disease (PD) at the evaluation time, respectively. We observed that miR-939 showed a negative correlation with chemotherapy response in our enrolled cases, in which low expression of miR-939 was observed more frequently in NC + PD subset (41/56, 73.2%) than in CR + PR set (15/56, 26.8%) (*P* < 0.001, Table 1). Moreover, Receiver operating characteristic (ROC) curves analysis demonstrated that a promising predictive value of miR-939 regarding GC chemotherapy response (area under the curve [AUC] =0.777, *P* < 0.001, Fig. 1d).

**Table 1:** Correlation between the expression of miR-939 and therapy response in GC patients (*N* = 110)

		miR-939 expression level		
	All cases	Low expression	High expression	*P* value
Therapy response				
CR + PR	57	15	42	
NC + PD	53	41	12	*P* < 0.001

*CR* complete response, *PR* partial response, *NC* no change, *PD* progressive disease

### miR-939 inhibits the GC growth in vitro and in vivo

Next, we investigated the effects of miR-939 on GC by overexpressing or inhibiting miR-939 in GC cell lines. MTT and colony formation assays revealed that overexpression of miR-939 significantly increased the growth rate of both GC cell lines; conversely, depletion of miR-939 promoted GC cell proliferation and tumorigenicity in vitro (Fig. 1e, f). Next, we sought to determine whether miR-939 sensitized GC cells to 5-Fu treatment, the common used chemotherapeutic drug in GC patients. As shown in Fig. 2a, b, the combination of 5-Fu with miR-939 was more efficient in reducing the GC cell viability and the clone formation ability. We further examined whether miR-939 increased the sensitivity of GC cells to 5-Fu by enhancing the rate of apoptosis. The AnnexinV-PI assay showed that miR-939-overexpressing cells displayed increased cellular apoptosis and necrosis in response to 5-Fu treatment at 48 h (Fig. 2c). Moreover, a significant increase in level of cleaved caspase-3 and PARP I in miR-939-overexpressing cells treated with 5-Fu was detected by western blot analysis (Fig. 2d). Together, these results demonstrate that miR-939 promoted the apoptosis of GC cells.

**Fig. 2:** miR-939 increases cellular sensitivity to 5-Fu in vitro and in vivo. **a** concentration-dependent growth inhibition in response to 5-Fu in miR-939-overexpressing, miR-939-silenced, and control GC cells. **b** quantification of the colony formation efficiency in miR-939-overexpressing, miR-939-silenced, and control GC cells treated with 5-Fu chemotherapy. **c** miR-939 sensitizes GC cells to 5-Fu-induced apoptosis. miR-939-overexpressing and vector control cells treated with indicated dose of 5-Fu for 24 h. Cell apoptotic death events were monitored by Annexin V/PI staining and flow cytometry assays. **d** after treatment, cleaved caspase 3 and PARP levels were determined by western blot, and GAPDH was used as a normalized control. The quantitative values under the bands were the relative ratios cleaved PARP, cleaved caspase-3 to GAPDH from densitometric analysis. **e** the same amount (3x10^6^) of miR-939-overexpressing and control GC cells were injected subcutaneously into the flanks of nude mice. Starting on day 7, the mice were given 5-Fu or DMSO intraperitoneally. **f**, **g** and **h** the tumor volumes (**f**) and mice weight (**h**) were monitored on day 7 and then every 2 days, as indicated, and the xenografts were excised and weighed on day 25 (g). *P < 0.05, ** *P* < 0.01

We also demonstrated miR-939’s ability to inhibit the GC growth using GC orthotropic animal model in vivo. As shown in Fig. 2e, we found that overexpression of miR-939 could significantly compromise GC tumor growth in vivo, and moreover, the combination of miR-939 and 5-Fu showed more significant inhibition of tumor growth, compared to either miR-939 or 5-Fu alone. Similarly in Fig. 2f, g, the group receiving combination of miR-939 and 5-Fu had lower average tumor weight and volume, compared with the groups receiving miR-939 or 5-Fu alone. More importantly, the combination of miR-939 and 5-Fu is well tolerated by the test animals in vivo, as indicated by mouse body weight (Fig. 2h). Thus, results suggested that miR-939 could enhance the sensitivity of GC cells to chemotherapies in vivo.

### miR-939 inhibits GC cell metastasis in vitro and in vivo

As lower expression of miR-939 was observed in patients with distant metastasis in GC, and distant metastasis often resulted in resistance to the conventional chemotherapy drugs, we sought to determine whether miR-939 has inhibition on GC metastasis. We confirmed that overexpression of miR-939 suppressed cellular migration and invasion, whereas miR-939 inhibition promoted migration and invasion in vitro (Fig. 3a-c). Moreover, we stained the cancer cells that spread into lung of mice. Number and size of the metastatic colonization were dramatically decreased on the lung surface of miR-939-transfected cells implanted mice compared to the control mice, and the miR-939 overexpression group exhibited much lower Ki-67 IHC staining of tumor metastases than the control group (Fig. 3d).

**Fig. 3:** miR-939 inhibits gastric cancer metastasis in vitro and in vivo. **a** the wound healing rate in miR-939-transfected cells was significantly inhibited, while accelerated in miR-939-silenced cells. **b** the number of migrated cell was decreased in miR-939-overexpressing, while increased in miR-939-silenced GC cells, as assessed by transwell migration assay. **c** the number of invaded cell was decreased in miR-939-overexpressing, while increased in miR-939-silenced GC cells, as assessed by Matrigel invasion assay. **d** miR-939 inhibits tumor metastasis in vivo. *Left panel*: hematoxylin and eosin (H&E) staining was performed on serial sections of metastatic tumors (M) and normal (N) lung. *Arrows*: lesions of lung. The Ki-67 IHC staining was performed on tumor metastases. *Right panel*: the number of nodules was qualified on lungs of SCID mice (*n* = 6 per group) 4 weeks after tail vein injection of SGC-7901-scramble (*left bars*) and SGC7901-miR-939 cells (*right bars*)

### miR-939 enhances GC chemosensitivity and inhibits metastasis by directly targeting SLC34A2

Using miRNA target prediction algorithms, we identified solute carrier family 34 member 2 (SLC34A2) as tentative target of miR-939 (Fig. 4a). The luciferase reporter assay indicated that overexpression of miR-939 significantly repressed the luciferase activity of SLC34A2-3’UTR, while inhibition of miR-939 increased the luciferase activity of SLC34A2-3’UTR. Meanwhile, ectopically expressing miR-939 mutation had no inhibitory effect on the SLC34A2-3’UTR luciferase activity (Fig. 4b). As shown in Fig. 4c, d, the expression levels of SLC34A2 mRNA and protein were significantly decreased following the ectopic expression of miR-939; In contrast, the inhibition of miR-939 led to an increase in the expression of SLC34A2 at both the mRNA and protein level. Consistently, overexpressing miR-939 mutation had no comprising effect on SLC34A2 mRNA and protein expression level (Fig. 4c, d). Moreover, our clinical data show that the expression levels of miR-939 and SLC34A2 were negatively correlated in 112 GC samples (r = −0.623, *P* < 0.001, Fig. 4e, f).

**Fig. 4:** SLC34A2 is the direct target of miR-939. **a** predicted miR-939 target sequence in 3'UTR of SLC34A2 (SLC34A2-3′UTR) and mutant containing three altered nucleotides in the seed sequence of miR-939 (miR-939-mut). **b** luciferase assay of pGL3-SLC34A2-3′-UTR reporters cotransfected with increasing amounts (10, 20, and 50 nM) of miR-939 mimic and mutant oligonucleotides in GC cell lines, or with increasing amounts (20, 50, and 100 nM) of miR-939 inhibitor oligonucleotides in GC cell line. **c** real-time RT-PCR analysis showed that overexpression of miR-939 significantly suppressed SLC34A2 mRNA expression level of SLC34A2 of GC cells, while inhibition of miR-939 led to a noticeable increase in SLC34A2 mRNA expression level of GC cell. **d** western blot analysis demonstrated that miR-939 tranfection decreased SLC34A2 protein level of GC cells, while anti-miR-939 dramatically increased SLC34A2 protein in GC cell. **e** high SLC34A2 IHC staining was observed in one GC sample with low miR-939 expression (*upper panel*); one GC sample with high miR-939 expression showed weak GNA13 IHC staining (*lower panel*). **f** the expression of SLC34A2 was inversely correlated with the expression of miR-939 in 112 GC samples. * *P* < 0.05, **P <0.001

To determine whether SLC34A2 directly contribute to miR-939 function, SLC34A2 was overexpressed in miR-939-overexpressing GC cells (Fig. 5a). As expected, restoration of SLC34A2 can block the miR-939-enhanced chemosensitivity and induction of apoptosis by 5-Fu treatment (Fig. 5b-d). Also, exogenously expressed SLC34A2 compromised the inhibition of metastasis by miR-939 on GC cells (Fig. 5e-f). Taken together, these data suggest that SLC34A2 played an important role for the effects of miR-939 on GC cells.

**Fig. 5:** Alteration of SLC34A2 levels influences the in vitro effects of miR-939 in GC cells. **a** protein levels of overexpressed SLC34A2 lacking 3'UTR in miR-939-overexpressing GC cells, as assessed by western blot. **b** and **c** MTT analysis (**b**) and colony formation assay (**c**) indicated that restoration of SLC34A2 in miR-939-overexpressing GC cells recovered cellular proliferation and tumorigenicity ability. **d** Annexin V/PI staining assays showed that restoration of SLC34A2 in miR-939-overexpressing GC cells decreased 5-Fu-induced apoptosis. **e** the migratory capacity of miR-939-overexpressing GC cells was enhanced after transfected with full-length SLC34A2, as assessed by a wound-healing assay. **f** overexpression of SLC34A2 in miR-939-transfected cells increased the number of invaded cell, as assessed by a Matrigel invasion assay. **g** in GC cells with miR-939 overexpression, the expression levels of p-ERK (*lane 2*) were significantly decreased compared with the control (*lane 1*). Restoration of SLC34A2 abrogated the decreased expression of p-ERK induced by miR-939 in GC cells (*lane 3*). Western blot analysis demonstrated that ERK inhibitor LY294002 (LY) could effectively decrease expressions of p-ERK induced by SLC34A2 (*lane 4*). **h** western blot analyses show that the expression of C-Raf and p-MEK was decreased in miR-939-transfected cells, while increased after SLC34A2 overexpressed

### miR-939 attenuates ERK1/2 phosphorylation and inhibits the Raf-MEK-ERK pathway

Previous studies have documented that PI3K/AKT and MAPK/ERK signaling pathway play crucial roles in development of chemoresistance and metastatic ability in human malignancies [14–16], thus we investigated the roles of miR-939 in the activation of PI3K/AKT and MAPK/ERK pathway. We found that the expression level of P-ERK was significantly decreased in cells with stable overexpression of miR-939 (Fig. 5g, lane 1, 2). This effect was reversed when we restored the SLC34A2 expression (Fig. 5g, lane 3). And pretreatment with ERK inhibitor U0126 could obviously reduce the expression level of P-ERK (Fig. 5g, lane 4). However, the P-AKT and AKT levels were not significantly altered. The observation that miR-939 compromised ERK1/2 activation leads us to further investigate the effect of miR-939 overexpression on RAS-RAF-MEK-ERK pathway. We found obvious inhibition of RAF-MEK-ERK pathway upon miR-939 overexpression, whereas restoration of SLC34A2 attenuated this compromising effect (Fig. 5h).

### Clinical significance and prognostic values of miR-939 and SLC34A2 in GC patients

We evaluated the prognostic significance of miR-939 and SLC34A2 protein expression levels in the GC patients who underwent surgery followed by chemotherapy. GC patients with high levels of miR-939 showed better overall survival (OS) rates and lower tumor recurrence rates than those with low miR-939 (Fig. 6a, b); whereas GC patients with high levels of SLC34A2 showed poorer OS rates and higher tumor recurrence rates than those with low SLC34A2 (Fig. 6c, d). According to univariate analysis, miR-939, SLC34A2 level, and TNM stage were significantly associated with OS and time to recurrence (TTR) in patients with GC (Table 2), while multivariate analysis confirmed miR-939, SLC34A2 level, and TNM stage as independent prognostic indicators for both OS and TTR (Table 2).

**Fig. 6:** The prognostic significance of miR-939 and SLC34A2 for 112 GC patients assessed by Kaplan-Meier analyses. **a** and **b** patients with higher miR-939 had (**a**) better overall survival (OS) and (**b**) lower possibility for tumor recurrence. **c** and **d** patients with higher SLC34A2 levels in GC tissues had (**c**) poorer OS and (**d**) higher probability of tumor recurrence. **e** and **f** patients in subgroup I had the (**e**) longest OS and (**f**) lowest possibility of tumor recurrence among the four subgroups, which were divided according to combinations of miR-939 and SLC34A2, i.e., I, high miR-939/low SLC34A2; II, high miR-939/high SLC34A2; III, low miR-939/low SLC34A2; IV, low miR-939/high SLC34A2. For each cohort, different subgroups were plotted according to the cut-off values of miR-939 and SLC34A2, which were defined as the median of the cohort

**Table 2:** Univariate and multivariate analysis of factors associated with overall survival and time to recurrence in GC patients

	Overall Survival		Time To Recurrence	
Clinical Variables	HR (95% CI)	*P* value	HR (95% CI)	*P* value
Univariate analysis				
miR-939 (high versus low)	0.122 (0.053–0.281)	<0.001	0.228 (0.121–0.429)	<0.001
SLC34A2 (high versus low)	4.555 (2.241–9.260)	<0.001	4.179 (2.247–7.769)	<0.001
Gender (female versus male)	0.559 (0.294–1.060)	0.075	0.791 (0.441–1.420)	0.433
Age (≥60 versus < 60 years)	1.188 (0.614–2.297)	0.609	1.063 (0.588–1.921)	0.839
T status (T4 versus T1 + 2 + 3)	2.242 (1.182–4.254)	0.013	1.837 (1.042–3.239)	0.035
N status (N2 + 3 versus N1 + 2)	6.324 (2.463–16.239)	<0.001	4.928 (2.301–10.555)	<0.001
Clinical stage (III versus II)	14.407 (3.461–59.972)	<0.001	9.070 (3.250–25.313)	<0.001
Tumor size (≥5 cm versus < 5 cm)	2.080 (1.097–3.947)	0.025	2.057 (1.164–3.631)	0.013
Tumor grade (G3 versus G1 + 2)	1.371 (0.667–2.828)	0.389	1.354 (0.716–2.560)	0.351
Combination of miR-939 and SLC34A2				
II versus I	3.482 (0.778–15.581)	0.103	2.776 (0.971–7.939)	0.057
III versus I	6.822 (1.801–25.842)	0.005	2.971 (1.074–8.219)	0.036
IV versus I	24.212 (7.049–83.161)	<0.001	11.118 (4.688–26.368)	<0.001
Multivariate analysis^a^				
miR-939 (high versus low)	0.167 (0.070–0.398)	<0.001	0.328 (0.168–0.640)	0.001
SLC34A2 (high versus low)	2.287 (1.050–4.981)	0.037	2.517 (1.276–4.965)	0.008
T status (T4 versus T1 + 2 + 3)	1.642 (0.833–3.233)	0.152	1.403 (0.776–2.533)	0.262
N status (N2 + 3 versus N1 + 2)	3.812 (1.426–10.188)	0.008	3.143 (1.418–6.966)	0.005
Tumor size (≥5 cm versus < 5 cm)	1.784 (0.929–3.425)	0.082	1.754 (0.982–3.133)	0.058
Multivariate analysis^b^				
Combination of miR-939 and SLC34A2				
II versus I	3.320 (0.734–15.015)	0.119	2.865 (0.980–8.376)	0.055
III versus I	7.988 (2.077–30.727)	0.003	3.444 (1.224–9.689)	0.019
IV versus I	15.959 (4.498–56.619)	<0.001	7.970 (3.249-19.546)	<0.001
T status (T4 versus T1 + 2 + 3)	1.697 (0.852–3.382)	0.133	1.423 (0.782–2.590)	0.249
N status (N2 + 3 versus N1 + 2)	3.862 (1.443–10.339)	0.007	3.157 (1.424–7.001)	0.005
Tumor size (≥5 cm versus < 5 cm)	1.833 (0.949–3.543)	0.071	1.789 (0.998–3.240)	0.055

Combination of miR-939 and SLC34A2: I, High miR-939 and Low SLC34A2; II High miR-939 and High SLC34A2; III Low miR-939 and Low SLC34A2; IV Low miR-939 and High SLC34A2

Analysis was conducted using univariate or multivariate Cox proportional hazards regression

^a^Multivariate analysis of miR-939, SLC34A2, T status, N status and Tumor size

^b^Multivariate analysis of the combination of miR-939 and SLC34A2, T status, N status and Tumor size

Next, we divided patients into four groups based on miR-939 and SLC34A2 expression levels. GC patients with high miR-939 and low SLC34A2 had the best OS, lowest TTR, and best prognosis. In contrast, those with low miR-939 and high SLC34A2 had the poorest prognosis with the lowest OS and highest probability of tumor recurrence (*P* < 0.001; Fig. 6e, f). The combination of miR-939 and SLC34A2 was an independent prognostic indicator for OS and TTR (*P* < 0.001, Table 2). This combination gave even better prognostic power than miR-939 or SLC34A2 alone.

## Discussion

In this study, we found that miR-939 was indeed downregulated in GC tissues. Importantly, we reported, for the first time, that levels of miR-939 were inversely correlated with local relapse, distant metastasis and chemoresistance in GC patients. In addition, a series of in vitro and in vivo experiments demonstrated that miR-939 diminishes GC cell chemoresistance and metastatic ability by targeting SLC34A2 expression, with consequent inhibition of the Raf-MEK-ERK signaling pathway.

Based on the fact that miRNAs are involved in the initiation and progression of a variety of cancer types, the therapeutic potential value of miRNAs in cancer has been identified. A few in vivo and preclinical studies have reported modulating miRNA expression for cancer treatment [17–19]. In general, the therapeutic modulation of miRNAs is achieved by inhibiting oncogenic miRNAs, or by reconstituting tumor suppressor miRNAs [20, 21]. To our knowledge, the relationship between miR-939 expression and clinical implication in human cancers has not been analyzed previously. Here, we reported that miR-939 could repress tumor metastasis and increase the sensitivity of tumor cells to chemotherapies in GC. Our results indicated, for the first time, that the combination of miR-939 and 5-Fu was more efficient in killing GC cells in vitro and in vivo than using miR-939 or 5-Fu alone. Besides, we provide comprehensive evidence at cellular levels and in the animal models that miR-939 may be beneficial for GC patients with high risks of tumor recurrence and metastasis. Thus, the examination of miR-939 expression could be applied as an effective additional tool to optimize clinical decisions, enabling clinicians to identify those high-risk GC patients with increased risk of tumor recurrence and/or metastasis. Based on these findings, modulating miR-939 expression in GC appears to be an encouraging prototype therapeutic agent for cancer therapy, which might generate suppressing effect on GC chemotherapy resistance and distance metastasis. In general, these data suggested that miR-939 has a pivotal function in GC pathogenesis, with possible use as a biomarker and intervention point for new therapeutic strategies.

Interestingly, while little is known about the role of miR-939 in human cancers, miR-939 is among a unique set of downregulated miRNAs in GC. On the other hand, however, Ying reported upregulation of miR-939 in human ovarian cancer, which promoted cancer cell proliferation [22]. By conducting the current study, we provide compelling biologic as well as clinical evidence that miR-939 plays a tumor suppressive role in human GC. These seemingly contradictory findings suggested a dual role of miR-939 as both a tumor-promoting and -suppressive miRNA, underscoring the need to define the specific role of a miRNA in a certain type of cancer. As miRNAs can play multiple roles by targeting different genes, it is possible that a single miRNA could function as both a tumor-promoting or -suppressive miRNA in different tumor types depending on the genes and/or pathways they affect [23–25]. Herein, it remains important to thoroughly understand the molecular mechanisms mediating the differential biologic effects and targets of miR-939 in GC and other cancer types. This also underscored the need to define the differential biologic effects and targets of miR-939 in GC and other cancer types.

As described above, miRNAs can play multiple roles by targeting different genes. In this study, we identified SLC34A2 as miR-939 target genes. The *SLC34A2* gene, located on chromosome 4p15.2, is a member of the solute carrier gene family, which mediate the transport of inorganic phosphate into epithelial cells via sodium ion co-transport [26, 27]. Recently, function analyses of SLC34A2 in tumorigenesis have yielded contradictory results in different cancer models. Elevated expression of SLC34A2 has been observed in thyroid cancer and breast cancer [28, 29], but a significantly decreased expression has been reported in non-small cell lung carcinomas tissues [29, 30]. However, the expression pattern and biological role of SLC34A2 in GC has never been reported. Our data indicate that the restoration of SLC34A2 blocked the miR-939 overexpression-induced inhibition of cancer growth, cell proliferation, metastasis, and the induction of apoptosis. In addition, our clinical data show that expression of SLC34A2 is inversely correlated with miR-939 expression, and that patients with high expression of SLC34A2 have a decreased survival rate. Theses data, combined together, implied a potential oncogenic role of SLC34A2 in GC tumor development and progression.

The Ras/MEK/ERK pathway is a central signaling component that plays vital role in the initiation and regulation of various cellular processes, including proliferation, differentiation, apoptosis and migration [31, 32]. In mitogen-stimulated cells, MEK1/2 activation is directly regulated by MAPKs, including Raf-1 kinase, which phosphorylates 2 serine residues (S218, S222) in the activation loop of MEK, and thus in turn activates ERK1/2 [33–35]. Numerous reports have shown the aberrant activation of Raf/MEK/ERK pathway in variety of human cancers [36, 37]. Recent studies also demonstrated aberrant regulation of this pathway was associated with cancer chemoresistance [14, 15]. In the present study, we observed that miR-939 overerxpression in GC cells significantly decreased MEK1/2 phosphorylation and Raf-1 level, while restoration of SLC34A2 rescued these effects. Taken together, these findings demonstrated that SLC34A2 is an integral mediator of miR-939 function in GC cells via MEK-ERK MAPK pathway inhibition, which is known to be dysregulated in many cancers. However, the mechanism by which miR-939-SLC34A2 activates the MAPK signaling pathway is under investigation in our laboratory currently.

## Conclusion

In summary, we provide comprehensive evidence of the inhibitory effect of miR-939 on GC metastasis, and suggest a critical role of miR-939 in enhancing GC cell’s sensitivities to 5-Fu based chemotherapy. Our findings strongly suggest that miR-939 could be used for the development of novel combinatorial therapy strategies aimed at overcoming chemo-resistance and compromising metastasis in GC.

## Additional file

Additional file 1: Table S1. The clinicopathologic characteristics of the 112 GC patients who received surgery followed by adjuvant chemotherapy in this study. (DOC 40 kb)

## Abbreviations

5-Fu: 5-fluorouracil
AUC: Area under the curve
CR: Complete response
FFPE: Formalin-fixed paraffin-embedded
GC: Gastric cancer
IHC: Immunohistochemical
NC: No change
OS: Overall survival
PD: Progressive disease
PR: Partial response
ROC: Receiver operating characteristic
TTR: Time to recurrence
